The article "Primary Squamous Cell Carcinoma in a Transplanted Kidney: A Unique Case Highlighting Challenges in Diagnosis and Management" was published in 2025. Journal: Cureus.

# Primary Squamous Cell Carcinoma in a Transplanted Kidney: A Unique Case Highlighting Challenges in Diagnosis and Management

**DOI:** 10.7759/cureus.77154

**Published:** 2025-01-08

**Authors:** Ricardo A Pagan Santini, Madhu Bhaskaran, Vinay Nair, Gayatri Nair, Ahmed Fahmy

**Affiliations:** 1 Department of Internal Medicine, Long Island Jewish Forest Hills, Northwell Health, New York, USA; 2 Department of Nephrology and Transplant Nephrology, Northwell Health, New York, USA; 3 Department of Nephrology, Division of Transplant Surgery, Northwell Health, New York, USA; 4 Department of Surgery, Division of Transplant Surgery, Northwell Health, New York, USA

**Keywords:** cancer surveillance, immuno suppression, nephrololgy, renal allograft, renal squamous cell carcinoma, renal transplant, squamous cell carcinoma (scc)

## Abstract

Kidney transplantation is the preferred treatment for end-stage renal disease, but it involves risks, including an increased chance of malignancy due to several variables. We present a rare case of primary renal squamous cell carcinoma (SCC) in an allograft kidney. This patient, who had a renal transplant one year prior, presented with oliguria, elevated creatinine, and asthenia. Imaging done raised suspicion of a mass-like structure and biopsy subsequently done confirmed a primary SCC in the transplanted kidney, leading to a total nephrectomy and hemodialysis initiation. This case highlights the different cancer risks faced by transplant recipients, particularly due to immunosuppressive medications. We discuss emerging alternatives in immunosuppression that may mitigate these risks. Given the rarity of primary SCC in allografts, determining the cancer’s origin whether primary or metastatic is critical for effective management since this distinction could shape future approaches to managing allograft malignancies. We also emphasize the importance of establishing imaging and monitoring guidelines and how combining imaging with serum and urine studies may enhance cancer surveillance, aiding in long-term graft health and transplant longevity.

## Introduction

Kidney transplants have become a critical area of research in nephrology over the past years since they are the preferred treatment for end-stage renal disease. However, transplants are still associated with persistent complications, one of the most concerning being malignancy. While skin cancers are the most reported post-transplant malignancies, there are rare occurrences of allograft tumors, such as renal cell carcinoma and papillomas originating within the kidney tissue itself [1]. In this report, we present a rare case of primary renal squamous cell carcinoma (SCC) occurring in an allograft kidney. Although risk factors contributing to renal SCC are well-documented, these cases have been identified in native kidneys rather than in transplanted organs, making this instance particularly unique [1]. Another significant factor contributing to malignancy in kidney transplant recipients is the lifelong use of immunosuppressive therapy. These medications are necessary to prevent organ rejection but come with the downside of increasing cancer risk [1]. This discussion will cover the mechanisms by which commonly used immunosuppressive drugs promote oncogenesis, as well as explore newer agents that aim to mitigate these risks while still being effective for transplant recipients. Additionally, we highlight the limitations of current screening guidelines, emphasizing opportunities to optimize these protocols for improved patient outcomes. Furthermore, we will explore how monitoring and screening methods from other types of SCCs might inform future strategies for malignancy detection and management in kidney transplant patients.

## Case presentation

A 58-year-old male patient, with a history of a right renal transplant one year and a half ago, previously on peritoneal dialysis secondary to diabetic nephropathy and a terminal creatinine of 2.7 mg/dL, hypertension, diabetes mellitus on insulin, kidney stones, and CMV viremia, presented to the emergency department with generalized weakness, decreased urine output, and dark urine. A week prior to presentation, he had been admitted for one week to the kidney transplant service for acute kidney injury suspected to be from COVID-19 infection versus CMV viremia which was treated with steroids and remdesivir. The patient while being in the hospital creatinine levels downtrended to baseline, urine output was adequate to weight, and the patient was discharged with outpatient follow-up. The patient noted that one day prior to the second admission, he started producing less urine with a darker color as well. The patient stated that he had been compliant with a home regimen of medications including immunosuppression medications which included CellCept, tacrolimus, and prednisone. Remarkable initial blood work done showed a creatinine of 3.01 mg/dL and a GFR of 23 ml/min/1.73 m^2^. The patient's initial laboratory results are shown in Table 1.

**Table 1:** Initial labs on day 1 of admission K/μL: thousands per microliter; g/dL: gram per deciliter; mmol/L: millimoles per liter; mg/dL: milligrams per deciliter; ml/min/1.73 m^2^: milliliters per minute per square meter; BUN: blood urea nitrogen; GFR: glomerular filtration rate

Labs	Results	Reference Ranges
White Blood Cell	4.06	3.80-10.50 K/μL
Hemoglobin	9.9	13.0- 17.0 g/dL
Platelets	336	150-400 K/μL
Sodium	134	135-145 mmol/L
Potassium	4.2	3.5-5.3 mmol/L
Chloride	98	96-108 mmol/L
BUN	61	7-23 mg/dL
Creatinine	3.01	0.50-1.30 mg/dL
GFR	23	>60 ml/min/1.73 m^2^

A renal ultrasound of the transplanted kidney was performed showing persistent urothelial thickening involving the renal collecting system and ureter with patent renal transplant vasculature. However, on color Doppler images, there could be diminished perfusion of the lower pole of the transplant along with tardus parvus waveform morphology. Also, there is a rounded area in the interpolar region of the transplanted kidney with uneven texture and slightly increased echogenicity compared to the surrounding cortex, possibly representing a renal mass. The findings described above are shown in Figure 1.

**Figure 1:** Renal ultrasound The figure depicts a focal rounded contour in the renal cortex which could represent a mass.

Due to concerns of impaired renal blood flow to the lower pole of the renal transplant, interventional radiology was consulted for a renal artery angiogram which was performed and did not reveal impaired blood flow in the renal vasculature. An MRI was also performed to clarify the renal mass. It showed a 4.4 cm by 8.2 lesion (Figure 2).

**Figure 2:** Abdominal MRI The figure depicts a non-contrast MRI showing the 4.4cm x 8.2 cm mass in the transplanted kidney.

Based on the above findings, interventional radiology was consulted to perform a renal biopsy, which revealed SCC with a histologic differentiation characteristic of primary renal origin (Figure 3 and Figure 4). During the hospitalization, the patient's serum creatinine continued to rise along with signs of fluid overload, for which the patient was started on intravenous diuretic therapy. Due to persistent symptoms along with worsening blood work and malignancy diagnosis, the patient required total nephrectomy which was performed along with initiation of hemodialysis. The patient is currently being followed with oncology and outpatient hemodialysis management.

**Figure 3:** Kidney biopsy sample with p63 staining confirming squamous cell carcinoma. Magnification used x40

**Figure 4:** Kidney biopsy sample with HMWK staining confirming squamous cell carcinoma. Magnification used x400 HMWK: High-molecular-weight cytokeratin

## Discussion

Primary renal SCC is an uncommon post-transplant malignancy. Even though the focus here is on allograft kidneys, it is crucial to recognize that native kidneys also remain susceptible to malignancy after transplantation. This increased risk is often linked to extended periods of dialysis, a condition whose underlying mechanisms are not fully understood but are thought to involve kidney inactivity, tubular hyperplasia, and cyst formation [1]. An essential step in managing renal malignancies in transplant patients is determining whether the malignancy originates from the allograft or is a metastatic lesion. Research suggests that tumors diagnosed within two years of transplantation are more likely to be primary allograft malignancies, whereas those detected after two years are considered metastatic disease [1]. Chronic inflammation has been an established underlying reason for developing primary renal SCC. Identified risk factors for SCC in native kidneys include recurrent urinary tract infections (with or without vesicoureteric reflux), long-standing staghorn calculi, smoking, exposure to schistosomiasis, exogenous and endogenous chemical exposure, vitamin A deficiency, and hormonal imbalances [1]. Although detailed mechanisms remain poorly understood due to the limited number of reported cases, it is believed that SCC of the urothelial tract develops through a process of metaplasia. Specifically, keratinizing squamous metaplasia of the urothelium is thought to significantly elevate the risk of developing SCC in the future [2]. The association between oncogenic viruses like Epstein-Barr virus (EBV) and cytomegalovirus (CMV) and renal cancer has been reported, particularly in cases involving high-grade tumors. Evidence suggests that these viruses contribute to cancer pathology by being present in tumor-infiltrating B cells, which may promote tumor development [2]. Additionally, other studies have indicated that EBV infection of renal proximal tubular cells might trigger a cellular immune response, leading to damage in the renal interstitium [2].

Chronic maintenance immunosuppression is another critical factor that predisposes post-transplant patients to malignancy. While a wide variety of immunosuppressive medications are available, all exert some degree of indirect oncogenic effect. For instance, calcineurin inhibitors promote oncogenesis, tumor growth, and metastasis by inhibiting DNA repair and apoptosis, while simultaneously stimulating the production of transforming growth factor-beta (TGF-beta) and vascular endothelial growth factor [3]. Azathioprine and its derivatives increase the risk of malignancy through enhanced DNA damage caused by ultraviolet (UV) exposure and the inhibition of DNA repair mechanisms [3]. The exact oncogenic mechanism of newer agents like mycophenolate mofetil remains unclear. However, it is known to reduce the production of guanosine nucleotides in both B and T lymphocytes, primarily affecting T cells, which may impair tumor recognition and immune response, contributing to oncogenesis [3]. Interestingly, it may be linked to reduced cancer incidence and nephrotoxicity, and some tumors regress if this medication is withdrawn [3]. This dilemma of balancing the dosage of immunosuppressants due to the high side-effect profiles highlights the need for an immunomodulatory approach rather than straightforward immunosuppression to optimize therapy while minimizing risks. 

Despite ongoing debate about transplanting kidneys with known malignancies, transplantation may provide significant mortality and morbidity benefits compared to dialysis, especially in elderly patients with multiple comorbidities who are not suitable candidates for healthy donor transplants [4]. This is true even in cases involving small tumors under 4 cm or those without capsular invasion [5]. When considering the transplantation of a kidney with a tumor, it is essential to assess how the malignancy may behave and evaluate how this may affect the patient. Research has shown that in some immunosuppressed patients who develop primary renal malignancies, there appears to be a degree of host resistance to tumor growth and spread [6]. Notably, the tumor grade plays a crucial role; low-grade tumors in immunosuppressed individuals often have shown similar linear growth patterns as in non-immunosuppressed patients [6]. This is interesting to note since in the past chronic antigenic stimulation in immunosuppressed patients enhanced tumor aggressiveness and metastatic potential. Determining the origin of the tumor cells is vital for appropriate management. Renal malignancies arising from the allograft kidney are classified as stage 1, where treatment options include partial nephrectomy, tumor resection, and ultrasound surveillance to preserve graft function [6]. Conversely, malignancies originating from host cells are considered stage 4, necessitating both native and transplant nephrectomy, a return to dialysis, and possibly chemotherapy [7]. This scenario renders the patient ineligible for another transplant for at least two years due to the risk of tumor recurrence [7]. Thus, identifying the tumor cell origin is imperative, highlighting the importance of prescreening to guide the optimal treatment plan.

Currently, the American Society of Transplantation has found insufficient evidence to recommend routine screening for primary renal malignancies in transplant recipients using ultrasound, computed tomography, or urine cytology [8]. However, there are patients at higher risk for these malignancies, and the absence of established screening guidelines means this population is often inadequately monitored. Ultrasound is generally favored for its accessibility, low cost, and noninvasive nature [8]. Nonetheless, it has limitations, particularly its insensitivity to small lesions, making it less effective for detecting early-stage disease [9]. Additionally, a significant concern when developing screening protocols is the risk of false positives from ultrasound, potentially leading to unnecessary biopsies and invasive procedures [9]. This is particularly problematic for immunocompromised patients, as these procedures can result in complications like bleeding, infections, graft dysfunction, or even graft loss [10]. Non-contrast computed tomography scans have been explored as an alternative due to their superior sensitivity and detailed imaging capabilities. However, the challenge of accurate tissue sampling remains unresolved, with unnecessary sampling carrying risks of harm and psychological distress for patients and their families [10].

Another important aspect of screening, monitoring, and guiding treatment for malignancies is the use of serum or urine tumor markers. While no specific marker has been identified for SCC of an allograft tumor, markers have proven helpful in other malignancies of squamous differentiation. For example, in cervical SCC, elevated levels of serum SCC antigen, hypersensitive C-reactive protein, and CA125 have been associated with recurrence [11]. Similarly, in esophageal SCC, serum levels of SCC antigen and albumin have been used to predict patient survival [11]. High levels of SCC antigen combined with low albumin are indicative of poorer outcomes [11]. Furthermore, measuring SCC antigen and other markers before and after treatment can help assess the patient’s response to therapy and provide insights into prognosis.

## Conclusions

Primary renal SCC is a rare but concerning complication in transplant recipients, likely due to several risk factors. Although there is limited data on the specific pathophysiology of SCC in renal allografts, existing knowledge about risk factors for SCC in native kidneys provides a foundation for understanding how this malignancy may emerge in transplant settings. A key modifiable risk factor for renal malignancies in transplant recipients is the use of immunosuppressive medications. These drugs are essential to prevent graft rejection but can also contribute to harmful side effects such as rejection of such and emphasize the need for new strategies of immunomodulation with a focus in beneficial long-term health outcomes. Another challenge in managing renal transplant-associated malignancies is differentiating between primary and metastatic tumors. Factors such as tumor size, location, and the timeframe since transplantation can help guide diagnosis and treatment decisions. Contributing to this issue is the lack of post-transplant cancer screening guidelines. Although recurrent imaging techniques like ultrasound and CT scans have been suggested, studies have not shown a clear benefit in reducing recurrence rates and potentially arising complications. A promising area for improvement lies in the use of serum and urine markers, which have shown success in detecting other squamous-origin malignancies. Integrating these markers with imaging may enhance early detection of primary tumors in allograft kidneys, leading to better outcomes for transplant recipients. Despite advancements in transplantation, developing comprehensive protocols for cancer surveillance and long-term organ viability remains essential to improve patient outcomes and quality of life.
